# Acetylbritannilactone attenuates contrast-induced acute kidney injury through its anti-pyroptosis effects

**DOI:** 10.1042/BSR20193253

**Published:** 2020-02-18

**Authors:** Fei Chen, Jingchao Lu, Xiuchun Yang, Bing Xiao, Huiqiang Chen, Weina Pei, Yaqiong Jin, Mengxiao Wang, Yue Li, Jie Zhang, Fan Liu, Guoqiang Gu, Wei Cui

**Affiliations:** Department of Cardiology, The Second Hospital of Hebei Medical University and The Institute of Cardiocerebrovascular Disease of Hebei Province, Shijiazhuang 050000, China

**Keywords:** Acetylbritannilactone, acute kidney injury, Contrast media, pyroptosis

## Abstract

Contrast-induced acute kidney injury (CI-AKI) is a severe complication caused by intravascular applied radial contrast media (CM). Pyroptosis is a lytic type of cell death inherently associated with inflammation response and the secretion of pro-inflammatory cytokines following caspase-1 activation. The aim of the present study was to investigate the protective effects of acetylbritannilactone (ABL) on iopromide (IOP)-induced acute renal failure and reveal the underlying mechanism. *In vivo* and *in vitro*, IOP treatment caused renal damage and elevated the caspase-1 (+) propidium iodide (PI) (+) cell count, interleukin (IL)-1β and IL-18 levels, lactate dehydrogenase (LDH) release, and the relative expression of nucleotide-binding domain, leucine-rich repeat containing protein 3 (NLRP3), apoptosis-associated speck-like protein (ASC), and gasdermin D (GSDMD), suggesting that IOP induces AKI via the activation of pyroptosis. Furthermore, the pretreatment of ABL partly mitigated the CI-AKI, development of pyroptosis, and subsequent kidney inflammation. These data revealed that ABL partially prevents renal dysfunction and reduces pyroptosis in CI-AKI, which may provide a therapeutic target for the treatment of CM-induced AKI.

## Introduction

In recent years, vascular administration of iodinated contrast media (CM) has been widely used in patients undergoing diagnostic cardiac angiography and percutaneous coronary intervention [1]. Contrast-induced acute kidney injury (CI-AKI) occurs in more than 5–15% of patients after percutaneous coronary intervention via CM [2], which is associated with risk factors, such as advanced age, diabetes, and hypertension [3]. CI-AKI is the third most common cause of acute renal failure in hospitalized patients after hypoperfusion and nephrotoxic drugs [4]. A previous study showed that CI-AKI is associated with major adverse clinical outcomes and death [5]. Once CI-AKI occurs, there is no specific treatment; hence, prevention by minimizing contrast administration and Intravenous (IV) fluid hydration is the optimal management strategy [6]. However, clinical data regarding their feasibility, efficacy, and safety are limited [7]. Multiple adjunctive pharmacotherapies for CI-AKI prevention have been tested. For example, N-acetylcysteine (NAC) was reported to reduce the risk of CI-AKI by reactive oxygen species scavenging [8]. However, PRESERVE and acetylcysteine (ACT) trials failed to indicate a decline in adverse renal outcomes with oral NAC. Similarly, the effect of renin–angiotensin–aldosterone inhibitor in CI-AKI is contradictory [9]. It is therefore urgent to explore the pathological mechanisms of CI-AKI for effective treatment.

Pyroptosis is a unique type of programmed cell death that is distinct from apoptosis and necrosis [10]. Pyroptosis is a pro-inflammatory response and depends on the activation of the caspase cascade and interleukin (IL) cytokine family members [11]. Nucleotide-binding domain, leucine-rich repeat containing protein 3 (NLRP3) recruits apoptosis-associated speck-like protein (ASC) and pro-caspase-1 to form an NLRP3 inflammasome, which induces the release of inflammatory cytokines IL-1β and IL-18 [12]. The release of mature IL-1β and IL-18 in conjunction with inflammasome-driven cell death is termed as pyroptosis [13]. In addition, caspase-1 drives pyroptosis via activation of the pore-forming protein gasdermin D (GSDMD) [14]. Some reports showed that pyroptosis is triggered by a variety of pathological stimuli, including myocardial infarction, stroke, and malignancy [15–16]. AKI was associated with increased levels of pro-inflammatory cytokines and manifested by pyroptosis [17]. A previous study showed that caspase 4/5/11-mediated pyroptosis is required for the activation of CI-AKI [18], which reflects the positive correlation between pyroptosis and CI-AKI. Thus, controlling the progress of pyroptosis might provide new insight into CI-AKI therapy.

Acetylbritannilactone (ABL) is a new active extract from a traditional Chinese medicinal herb, *Inula britannica* [19]. Previous studies have indicated that ABL has antioxidant, anti-inflammatory, and organ-protective activities *in vivo* and *in vitro* [20–21]. ABL prevented acute renal injury by inhibiting apoptosis and alleviating inflammation and oxidative stress in exhaustive swimming rats [22]. However, the effect of ABL on CI-AKI is unknown.

In our study, we found that the treatment of iopromide (IOP) into human kidney cells (HK-2) significantly up-regulated the levels of IL-1β and IL-18, lactate dehydrogenase (LDH) release activity, and the expression of NLRP3, ASC, cleaved caspase-1, mature GSDMD, and IL-1β, indicating that IOP induced pyroptosis *in vitro. In vivo*, the application of IOP induced pyroptosis and resulted in acute kidney damage. The pretreatment of ABL partly blocked the levels of IL-1β and IL-18, LDH release activity, and the expression of NLRP3, ASC, cleaved caspase-1, mature-GSDMD, and IL-1β and restored kidney function damaged by IOP. These findings indicate that the application of iodinated CM induced AKI via the activation of pyroptosis, and the application of ABL partly reversed renal dysfunction in CM-injured mice kidneys via the blockage of pyroptosis. These data provided new evidence that ABL administration might be potential future therapeutic avenues to limit CM-associated AKI.

## Materials and methods

### Cell culture

HK-2 cell, a human kidney tubular epithelial cell line derived from a normal kidney, was obtained from American Type Culture Collection (ATCC, Manassas, VA). HK-2 cell was cultured in keratinocyte serum-free medium supplemented with bovine pituitary extract and human recombinant epidermal growth factor in a humidified atmosphere at 37°C with 5% CO_2_.

### Pyroptosis determination by flow cytometry assay

Pyroptosis was analyzed through flow cytometry (FACSCalibur; Becton Dickinson, Sunnyvale, CA) using the FAM Fluorochrome-labeled inhibitors of Caspases (FLICA) Caspase Assays kits (ImmunoChemistry Technologies, LLC, U.S.A.) according to the manufacturer’s instructions. HK-2 cells were treated with different drugs. Approximately 290 μl of cells at 3 × 10^5^ cells/ml were transferred into fresh tubes and stained with 10 μl of 30× FLICA buffer. After 30 min in the dark at 37°C, cells were treated with propidium iodide (PI) at the final concentration of 1 μg/ml and incubated in the dark for 5 min. Fluorescence intensity was quantified using a flow cytometry.

### Cell viability assay

HK-2 cells were seeded into 96-well culture plates at the density of 2000 cells/well. To determine the effect of different IOP concentrations (Ultravist 370, Bayer HealthCare LLC, Leverkusen, Germany) on cell viability, cells were seeded into six-well plates and incubated with IOP at the concentration of 0, 20, 40, 80, or 160 mg I/ml. After 2 h, cells were collected for Cell Counting Kit-8 (CCK-8) assay. To explore the effect of treatment time of IOP on cell viability, HK-2 cells were incubated with IOP at the concentration of 80 mg I/ml for 0, 10, 30, 60, or 120 min. When the density reached 80%, cells were incubated with 10 μl of CCK-8 reagent (Dojindo, Kumamoto, Japan) for 2 h at 37°C. The color reaction was measured at the wavelength of 450 nm with a SpectraMax Paradigm Multi-Mode Microplate Reader (Molecular Devices, Sunnyvale, CA). Each sample was repeated in triplicate.

### Enzyme-linked immunosorbent assay

The levels of IL-1β and IL-18 in HK-2 cells were assessed by human IL-1β and IL-18 Enzyme-linked immunosorbent assay (ELISA) Kit (Invitrogen, U.S.A.). The levels of mouse serum IL-1β and IL-18 were measured by mouse IL-18 and IL-1β ELISA Kit (Invitrogen, U.S.A.).

### LDH release assay

LDH release was measured using LDH Cytotoxicity Assay Kit (Beyotime, Beijing, China) according to the manufacturer’s instructions. LDH release was determined with a coupled enzymatic reaction that resulted in the conversion of a tetrazolium salt into a red color formazan by diaphorase. Cells were seeded into 96-well plates. When the density reached 80–90%, cells were treated with different drugs at different schedules. Then 120 μl of culture medium was transferred into a new 96-well plate and mixed with 60 μl of LDH work buffer. After 30 min in the dark at room temperature, the absorbance (Optical density, OD) was measured at the wavelength of 490 nm. The percentage of LDH release was calculated according to the following formula: percentage of LDH release = (OD_experimental group_ − OD_control group_)/(OD_max_ − OD_control group_) × 100%.

### Western blot

Renal tissue and cells were extracted using radio immunoprecipitation assay buffer (Sigma, U.S.A). The lysates were centrifuged and then supernatant was collected. Protein concentration in the supernatant was quantified by the bicinchoninic acid kit (ABP Biosciences, Wuhan, Hubei, China). The same amount of protein (40 μg/lane) was subjected into 12% sodium dodecyl sulfate/polyacrylamide gel electrophoresis (SDS/PAGE) and transferred to a polyvinylidene difluoride membrane (Millipore, Bedford, MA, U.S.A.). After being blocked by 5% nonfat milk in Tris-buffer saline (TBS) for 1 h, the membrane was probed with the following primary antibodies: rabbit monoclonal anti-NLRP3 (1:1000), anti-ASC (1:1000), anti-caspase-1 (1:500), anti-GSDMD (1:1000), and anti-glyceraldehyde 3-phosphate dehydrogenase (GAPDH) (1:2000, Cell Signaling Technology, Inc., Beverly, MA) antibodies and mouse monoclonal anti-IL-1β antibody (1:1000, Abcam, U.S.A.) overnight at 4°C. The next morning, the membrane was incubated with anti-rabbit IgG H&L (1:10000, Abcam, U.S.A.) for 2 h at 37°C. After TBST (TBS containing 0.05% Tween-20) washes, the blots were visualized with the enhanced chemiluminescence kit (Thermo Scientific, San Jose, CA, U.S.A.) and analyzed with ImageJ version 1.47i (U.S. National Institutes of Health, Bethesda, MD). The loading control was the constitutively expressed protein, GAPDH.

### Real-time reverse transcription polymerase chain reaction

Total RNA was isolated from kidneys of different groups using TRIzol reagent (Invitrogen, Carlsbad, CA). cDNA was synthesized using a PrimeScript RT Reagent Kit (Takara, Dalian, China). The real-time reverse transcription polymerase chain reaction (RT-PCR) used was a 2× One-Step SYBR Real-Time PCR Kit in an ABI 7500 system (Applied Biosystems Inc., Foster, CA) according to the manufacturer’s protocol. The parameters for RT-PCR were as follows: 95°C for 5 min, followed by 40 cycles of 94°C for 30 s and 60°C for 30 s. The relative expression level of target genes was normalized to the internal control GAPDH via the 2^−ΔΔ*C*_T_^ method. The primers for RT-PCR were as follows: NLRP3 forward primer: 5′-cgagacctctgggaaaaagct-3′, reverse primer: 5′-gcataccatagaggaatgtgatgtaca-3′; ASC forward: 5′-cttgtcaggggatgaactcaaaa-3′, reverse: 5′-gccatacgactccagatagtagc-3′; Caspase-1 forward: 5′-acaaggcacgggacctatg-3′, reverse: 5′-tcccagtcagtcctggaaatg-3′; GSDMD forward: 5′-gtgtgtcaacctgtctatcaagg-3′, reverse: 5′-catggcatcgtagaagtggaag-3′; IL-1β forward: 5′-tcgcagcagcacatcaacaagag-3′, reverse: 5′-ccacgggaaagacacaggtagct-3′; GAPDH forward: 5′-ggccgagaatgggaagcttgtca-3′, reverse: 5′-tcggcagaaggggcggagatga-3′. The experiments were conducted in triplicate with independent experimental samples.

### Animals and grouping

A total of 30 male C57BL/6 mice weighing 18–20 g (7–10 weeks of age) were purchased from Beijing Vital River Laboratory Animal Technology. All mice were housed in a facility with an alternating 12-h light/dark cycle at 20°C and 60% relative humidity and acclimated for 7 days before the experiments in Hebei Medical University. The mice were fed a commercial chow and allowed free access to water until 12 h before the experiments. All animal experiments were approved by the Animal Research Control Committee of Hebei Medical University. Mice were assigned randomly into five groups: control group (Cont, *n*=6), vehicle (Veh, *n*=6), ABL group (ABL, *n*=6), IOP group (*n*=6), and IOP + ABL group (*n*=6). IOP (Ultravist; 370 mg iodine/ml, 3.7 g iodine/kg; Bayer HealthCare LLC, Leverkusen, Germany) was used as the iodinated CM in the present study [23]. Mice in Cont or ABL group were given saline or ABL (25 mg/kg) via gavage administration for 6 days, respectively. Mice in IOP + ABL group were first gavage administered with ABL for 6 days. On the sixth day, mice in IOP and IOP + ABL groups were injected intraperitoneally with a prostaglandin synthesis inhibitor (indomethacin, 10 mg/kg; Sigma–Aldrich, St. Louis, MO, U.S.A.), a nitric oxide synthase inhibitor (NG-nitro-l-arginine methyl ester, 10 mg/kg; Sigma–Aldrich, St. Louis, MO, U.S.A.), and IOP (10 ml/kg). Mice in the Veh group were administered with the same amount of vehicle (methanol). On the seventh day, mice were anesthetized by intraperitoneal injection of pentobarbital sodium (30 mg/kg). Under anesthesia, the blood and kidney tissues from four groups were collected for follow-up experiments and following mice were killed using a lethal dose of pentobarbital sodium (100 mg/kg body weight).

### Kidney function

Blood samples were collected when animals were killed. Serum urea and creatinine concentrations were measured using an Olympus AU2700 analyzer (Diamond Diagnostics, Watford, U.K.).

### Hematoxylin and Eosin staining and tubular injury score

Renal tissues obtained from different groups were extracted and washed with phosphate-buffered saline (PBS), fixed in 10% formalin solution at 4°C overnight. After automated dehydration through a graded alcohol series, kidney slices were embedded in paraffin and cut into 5-μm sections. Sections were stained with Hematoxylin and Eosin (HE) and observed and captured using a light microscope (Nikon, Japan). All samples were evaluated by three investigators who are blinded to the experiment information. In HE sections, renal cortical vacuolization, peritubular/proximal tubule leukocyte infiltration, and proximal tubule simplification were evaluated and scored as follows: 0, normal; 1, mild injury; 2, moderate injury; and 3, severe injury. The tubule-interstitial injury score was defined as described previously [24].

### Statistical analysis

Data were expressed as the mean ± standard deviation (SD). Differences among different groups were analyzed by one-way analysis of variance (ANOVA) followed by multiple pairwise comparisons by the Newman–Keuls test using SPSS 17.0 software (SPSS Inc., Chicago, U.S.A.). *P*<0.05 was considered to be statistically significant.

## Results

### IOP-induced pyroptosis in HK-2 cells

To explore the effect of IOP on pyroptosis, we incubated HK-2 cells with IOP at different concentrations at various time intervals and performed flow cytometry. In Figure 1A,B, the percentage of caspase-1(+) PI (+) cells in total cells at 0 and 20 mg I/ml had no significant difference (*P*>0.05). However, the addition of IOP (40, 80, and 160 mg I/ml) significantly increased the percentage of caspase-1(+) PI (+) cells. Then we chose 80 mg I/ml for further experiments. As shown in Figure 1C,D, different incubation time of IOP had different effects on the percentage of caspase-1(+) PI (+) cells. With the extension of incubation time, the percentage of caspase-1(+) PI (+) cells significantly increased, except 10 min. In Figure 1E, CCK-8 assay revealed that 0 and 20 mg I/ml IOP had little effect on cell viability. Compared with the control group (0 mg I/ml), cell viability was significantly decreased after the treatment of 40, 80, and 160 mg I/ml IOP for 2 h. In Figure 1F, cell viability was obviously blocked after 30-, 60-, or 120-min incubation. In Figure 1G–J, the levels of IL-1β and IL-18 were significantly elevated after the incubation of IOP at 40–160 mg I/ml or for 30–120 min. Similarly, a significant increase in LDH release was observed after different IOP concentrations (40–160 mg I/ml) or various incubation periods (30–120 min), as shown in Figure 1K,L. These data indicated that IOP blocked cell viability, improved the levels of IL-1β and IL-18, and enhanced LDH release activity in dosage- and time-dependent manner.

**Figure 1:** IOP affected the percentage of caspase-1(+) PI (+) cells, cell viability, IL-1β levels, IL-18 levels, and LDH release activity in HK-2 cells in dosage- and time-dependent manner HK-2 cells were incubated with IOP at the concentration of 0–160 mg I/ml for 2 h. In addition, HK-2 cells were cultured with IOP at 80 mg I/ml for 0–120 min, respectively. Cells were collected for follow-up experiments. (**A**–**D**) The percentage of caspase-1(+) PI (+) cells was determined by flow cytometry. (**E,F**) Exhibited the effect of IOP on cell viability. (**G,H**) The IL-1β levels were examined by ELISA. (**I,J**) IL-18 levels were detected by ELISA. (**K,L**) Showed the effect of IOP on LDH release activity. *P<0.05, **P<0.01.

To further examine the relationship between IOP and pyroptosis, we incubated cells with IOP and examined the expression of key proteins for pyroptosis in Figure 2. In Figure 2A–F, the protein levels of NLRP3, ASC, cleaved caspase-1, and mature GSDMD were greatly improved after the incubation of IOP at 40–160 mg I/ml, and the expression of IL-1β was increased at 80 or 160 mg I/ml concentration. In Figure 2G–L, the levels of NLRP3, ASC, cleaved caspase-1, mature GSDMD, and IL-1β were significantly up-regulated after the incubation of IOP, except that mature GSDMD was decreased after 120 min. These data showed that IOP induced the expression of NLRP3, ASC, cleaved caspase-1, mature GSDMD, and IL-1β in dosage- and time-dependent manner. Taken together, we concluded that IOP induced pyroptosis in HK-2 cells.

**Figure 2:** IOP blocked the expression of proteins related to pyroptosis in dosage- and time-dependent ways (**A**) HK-2 cells were incubated with IOP at a concentration of 0–160 mg I/ml for 2 h, respectively. Proteins were extracted for Western blot. The relative expression of NLRP3 (**B**), ASC (**C**), cleaved caspase-1 (**D**), mature GSDMD (**E**), and IL-1β (**F**) was normalized to GAPDH. (**G**) HK-2 cells were incubated with IOP (80 mg I/ml) for 0–120 min, respectively. Proteins were isolated for Western blot. The relative expression of NLRP3 (**H**), ASC (**I**), cleaved caspase-1 (**J**), mature GSDMD (**K**), and IL-1β (**L**) was calculated by the normalization to GAPDH. *P<0.05, **P<0.01.

### ABL attenuates IOP-induced pyroptosis in HK-2 cells

To examine the effect of ABL on IOP-induced cells, we preincubated HK-2 cells with ABL for 2 h and then cultured cells with IOP. As shown in Figure 3A,B, there was no significant difference on the percentage of caspase-1(+) PI (+) cells between the control and ABL groups. The addition of only IOP enhanced the percentage; however, the pretreatment of ABL before IOP addition significantly blocked the up-regulation of the percentage induced by IOP. In Figure 3C, ABL greatly mitigated the cell viability blocked by IOP. In contrast, the IL-1β and IL-18 levels in the IOP group were enhanced than those in the control group, but the application of ABL blocked the up-regulation (Figure 3D,E). A similar trend was observed in LDH release activity (Figure 3F) and the mRNA and protein levels of NLRP3, ASC, caspase-1, GSDMD, and IL-1β (Figure 3G–Q). These data indicated that ABL conferred cytoprotection against IOP-induced pyroptosis in HK-2 cells.

**Figure 3:** ABL partly mitigated the effect of IOP on HK-2 cells HK-2 cells were randomly divided into four groups: control, ABL, IOP, and ABL + IOP groups. Cells in the ABL + IOP group were pretreated with ABL (100 μM) for 2 h and then incubated with IOP (80 mg I/ml) for 1 h. Cells in ABL or IOP groups were given ABL for 2 h or IOP for 1 h, respectively. The control group was administered with the same amount of vehicle. (**A,B**) The percentage of caspase-1 (+) PI (+) cells of four groups was determined by flow cytometry. (**C**) Cell viability was examined by CCK-8 kits. (**D,E**) IL-1β and IL-18 levels were detected by ELISA kits. (**F**) Shows the LDH release activity of the four groups. (**G**–**Q**) Protein or total RNA was extracted for Western blot or RT-PCR. The protein levels of NLRP3, ASC, caspase-1, GSDMD, and IL-1β were normalized to GAPDH. The mRNA levels of NLRP3, ASC, caspase-1, GSDMD, and IL-1β were normalized to GAPDH. Compared with the control group, ^a^*P*<0.01 and ^b^*P*<0.01 in the ABL+IOP group vs IOP group.

### ABL mitigated IOP-induced AKI via its anti-pyroptosis effects

We further detected the effect of ABL and IOP on mouse kidneys. We first determined the occurrence of IOP-induced AKI according to the levels of serum creatinine and urea. In Figure 4A,B, no significant difference on the levels of serum creatinine and urea was observed among Cont, Veh, and ABL groups. The levels of both serum creatinine and urea in IOP-injected mice were significantly up-regulated than those in the control group. However, the preinjection of ABL obviously reduced the serum creatinine and urea levels induced by IOP. In histological findings (Figure 4C), Cont, Veh, and ABL groups showed normal renal histology. The kidneys from IOP-injected mice exhibited an increase in kidney weight/body weight, brush border loss, and vacuolization in renal tubules displayed in Figure 4D,E. However, the application of ABL significantly alleviated the above symptoms. These data showed that IOP injection induced AKI, and ABL partly mitigated IOP-induced AKI.

**Figure 4:** ABL partly mitigated IOP-induced AKI via suppressing pyroptosis Mice were assigned randomly into five groups: control group (Cont, *n*=6), vehicle group (Veh, *n*=6), ABL group (ABL, *n*=6), IOP group (*n*=6), and ABL + IOP group (*n*=6). Mice in the Cont or ABL group were given saline or ABL (25 mg/kg) via gavage administration for 6 days, respectively. Mice in the IOP + ABL group were first gavage administered with ABL for 6 days. On the sixth day, mice in IOP and IOP + ABL groups were injected intraperitoneally with indomethacin, NG-nitro-l-arginine methyl ester, and IOP. Mice in the Veh group were administered with the same amount of vehicle (methanol). (**A,B**) Serum creatinine and urea levels were determined by ELISA. (**C**) Kidney tissues were extracted for HE stain. Scale bar = 100 μm. (**D,E**) show the kidney weight/body weight (%) and tubular injury score. (**F,G**) Serum IL-18 and IL-1β levels were determined by ELISA. (**H**) exhibits the LDH release activity. (**I**) Proteins were extracted for Western blot. (**J**–**N**) The relative protein levels of NLRP3, ASC, cleaved caspase-1, mature GSDMD, and IL-1β were normalized to GAPDH. (**O**) Schema depicting the mechanisms for renoprotection by ABL against IOP-induced AKI. *In vivo* and *in vitro*, the application of IOP significantly up-regulated the expression of NLRP3, caspase-1, ASC, and mature GSDMD, in turn promoting the release of pro-inflammatory cytokines IL-1β and IL-18 to induce pyroptosis and AKI. However, the pretreatment of ABL partly reversed the pyroptosis gene alterations in IOP-injured kidney and ameliorated AKI.

A previous study showed that IOP induced AKI via the activation of pyroptosis. In order to explore the mechanism by which ABL mitigated IOP-induced AKI, we first examined the levels of pro-inflammatory cytokines IL-18 and IL-1β. In Figure 4F,G, the serum IL-18 and IL-1β levels in the IOP group were significantly increased than those in the control group, and there was no obvious difference among the Cont, Veh, and ABL groups. However, the preinjection of ABL blocked the up-regulation of IL-18 and IL-1β induced by IOP. Similar results were found in LDH release activity. We also detected the protein levels of genes related to pyroptosis, including NLRP3, ASC, caspase-1, GSDMD, and IL-1β. As shown in Figure 4I–N, no significant difference was observed among the Cont, Veh, and ABL groups on the expression of NLRP3, ASC, cleaved caspase-1, mature GSDMD, and IL-1β, and the injection of only IOP significantly enhanced the protein levels of the aforementioned genes. However, after being challenged with IOP and ABL, HK-2 cells exhibited reduced NLRP3, ASC, cleaved caspase-1, mature GSDMD, and IL-1β expression, indicating ABL-mediated cytoprotection. These data showed that IOP caused AKI via the activation of pyroptosis, and ABL partly mitigated IOP-induced AKI via suppressing the activation of pyroptosis by IOP induction (Figure 4O).

## Discussion

AKI is a common and severe condition induced by various stimuli with a high mortality [25]. Iodinated CM-induced AKI accounts for 11% of cases of AKI and is the third most common cause of high morbidity and mortality in hospitalized patients [26]. Recent progress in interventional therapy and angiography has revived interest in explaining detailed mechanisms and developing effective treatment [27]. In our study, we investigated pyroptosis-related alterations that occur in renal tissues and renal tubule epithelial cells following IOP-induced AKI, suggesting that pyroptosis is a key event during CI-AKI. And we further determined the effect of ABL on IOP-induced AKI. We concluded that ABL exerts protective effects on CM-induced AKI via its anti-pyroptosis function. These findings revealed the mechanism by which CM induced AKI and provided new strategies for CM-induced AKI.

Pyroptosis is characterized by caspase-1-dependent formation of plasma membrane pores, leading to the release of pro-inflammatory cytokines [28]. Pyroptosis is closely associated with the activation of the NLRP3 inflammasome [29], which is a multimeric protein complex with ASC and pro-caspase-1 that leads to activation of caspase-1 [30–31]. Activated caspase-1 induces pyroptosis via the cleavage of GSDMD [32], which is a critical effector of pyroptosis [33–34]. Release of inflammatory cytokines such as IL-1β and IL-18 is the main feature of pyroptosis [35]. In our study, we found that the exposure of IOP to HK-2 cells is associated with an increase in the percentage of caspase-1 (+) PI (+) cells, IL-1β and IL-18 levels, LDH release activity, and the relative expression of NLRP3, ASC, caspase-1, GSDMD, and IL-1β. These data suggested the presence of IOP-induced pyroptosis in renal cells. In *in vivo* experiments, we found that the injection of IOP caused severe kidney morphological changes and increased the kidney weight/ body weight (KW/BW) percentage and tubular injury score, suggesting that IOP injection resulted in kidney function damage. In addition, the injection of IOP into mouse also increased the percentage of caspase-1 (+) PI (+) cells, IL-1β and IL-18 levels, LDH release activity, and the relative expression of NLRP3, ASC, caspase-1, GSDMD, and IL-1β. A previous study reported that caspase-11-mediated pyroptosis is closely related with Lipopolysaccharides (LPS)-induced septic AKI [36–37]. It is also reported that kidney epithelial pyroptosis played requisite roles in CI-AKI [38]. Combined with the previous study, we concluded that CM induced AKI via the activation of pyroptosis. These results provided new evidence that CM induced AKI and indicated the mechanism of CI-AKI.

ABL is a new active extract from a traditional Chinese medicinal herb. Some reports showed that ABL is widely used for treatments of cancers [39–40] and oxidative stress-related human diseases [41]. Only one report referred to the protective effects of ABL on exhaustive swimming exercise causing AKI [22]. In our study, we found that the pretreatment of ABL on IOP-injected mouse partially restored kidney function. Furthermore, ABL treatment partly blocked the up-regulation of the percentage of caspase-1 (+) PI (+) cells, IL-1β and IL-18 levels, LDH release activity, and the relative expression of NLRP3, ASC, caspase-1, GSDMD, and IL-1β induced by IOP in HK-2 cells and IOP-injected mouse, suggesting that ABL blocked IOP-induced pyroptosis. These data suggest that CM-induced AKI is partially due to cell pyroptosis, and such injury may be prevented by ABL administration.

In summary, our results suggest that CM induces AKI via the activation of pyroptosis, and the administration of ABL can alleviate CI-AKI through its anti-pyroptosis effects. These findings indicate that ABL might be a potential therapeutic agent for CI-AKI. However, there were some limitations in the study. First, although we found that CM induces AKI via the activation of pyroptosis, the mechanism by which CM mediates pyroptosis remains unclear. Could CM be involved in the activation of NLRP3 inflammasome, or the activation of caspase-1, or the cleavage of GSDMD? Second, we found that ABL alleviated CI-AKI via its anti-pyroptosis effects. However, the mechanism by which ABL was involved in the process of pyroptosis remains elusive. Third, our study was mainly focused on the effect of ABL in HK-2 cells and mice. But the clinical outcome of ABL was unknown. Therefore, further experiments need to be carried out in the future.

## Abbreviations

ABL: acetylbritannilactone
ACT: acetylcysteine
ASC: apoptosis-associated speck-like protein
CCK-8: Cell Counting Kit-8
CI-AKI: contrast-induced acute kidney injury
CM: contrast media
ELISA: enzyme-linked immunosorbent assay
FLICA: Fluorochrome-labeled inhibitors of Caspases
GAPDH: glyceraldehyde 3-phosphate dehydrogenase
GSDMD: gasdermin D
HE: Hematoxylin and Eosin
HK-2: human kidney-2
IL: interleukin
IOP: iopromide
IV: Intravenous
KW/BW: Kidney weight/body weight
LDH: lactate dehydrogenase
LPS: Lipopolysaccharides
NAC: N-acetylcysteine
NLRP3: nucleotide-binding domain, leucine-rich repeat containing protein 3
OD: Optical density
PI: propidium iodide
RT-PCR: real-time reverse transcription polymerase chain reaction
TBS: Tris-buffer saline
